RETRACTED

# Pan-Cancer Analysis of Prognostic and Immune Infiltrates for the TMEM65, Especially for the Breast Cancer

**DOI:** 10.1155/2023/9349494

**Published:** 2023-04-17

**Authors:** Xinming Song, Pintian Wang, Ruiling Feng, Mandika Chetry, E Li, Xiaohua Wu, Zewa Liu, Shasha Liao, Jing Lin

**Affiliations:** ^1^Department of Oncology, The First Affiliated Hospital of Shantou University Medical College, Shantou 515041, Guangdong, China; ^2^Department of Oncology, Shantou Longhu People's Hospital, Shantou, Guangdong, China

## Abstract

**Introduction:**

Transmembrane protein 65 (TMEM65) is an inner mitochondrial membrane protein, which played important role in mediating autophagy, smooth muscle contraction, protein glycosylation, and immune response. In recent years, the interest had risen for exploring the function of the TMEM genes in the cancer fields. As a consequence, in our pan-cancer research of the TMEM65, we explored the function of the gene in kinds of database and tried to apply the finding in the clinical practice.

**Methods:**

In this research, we provide a comprehensive investigation of TMEM65 expression in a pan-cancer manner containing 33 cancer types. We evaluated the association of TMEM65 with the prognosis, immune infiltration, drug sensitivity analysis, GSVA enrichment analysis, TMB, MSI, NEO, and hotspot mechanisms.

**Results:**

TMEM65 was abnormally expressed in 24 types of cancers and showed correlation with the OS for 6 cancers and PFI for 9 cancers and kpI for 3 types. Moreover, the TME score, CD8 T effector, and immune checkpoint scoring systems showed a close correlation with the TMEM65. Moreover, TMEM65 was strongly correlated with some of the most common tumor-related genes and certain pathways (TGF beta signaling, TNFA signaling, hypoxia, pyroptosis, DNA repairing, autophagy, ferroptosis, and other related genes). Additionally, the TMEM65 showed correlations with the tumor mutational burden (TMB), microsatellite instability (MSI), NEO, and drug sensitivity. Finally, we confirmed several pathways by the GSEA and GSVA for the TMEM65 at the breast cancer aspects. Nomogram prediction model was also established for the breast tumors based on the TMEM65 level and other variables.

**Conclusion:**

Above all, the TMEM65 played important roles in predicting the prognosis of the cancers and correlated with the tumor immunity in the pan-cancer analysis.

## 1. Introduction

Globally, cancer is the second leading cause of death. Clinicians and researchers are trying their best to find the target and markers to improve the prognosis of cancer. The pan-cancer analysis has recently emerged and acts as a new strategy to decern varieties of gene with potential predictability, by analyzing the data and pathways obtained from the TCGA, GEO, and Oncomine database. The researchers could find genes, pathways, or special RNAs with vital implications for the development, TME, immune-related, and other mechanisms for the cancers. The pan-cancer analysis played vital roles and shed light on distinguishing the complex relationship of the mechanism for the cancers. Recently, the pan-cancer analysis was conducted for the genes which represented the marker of the pyroptosis and the results showed strong evidence that the gene not only showed strong correlation with the prognosis but also the immune checkpoints and immune cells [1].

RETRACTED

Breast cancer is the leading cause of death in women worldwide. It has now experienced tremendous advances in fields of exploring potential prognosis markers. In spite of the fact that the pan-cancer analysis and other analyses (single cells, proteomics, and metabonomics) had made tremendous advances, most of the breast tumor patients suffer early and even late recurrence. Only a proportion of the ER-positive patients had successfully owned a complete remission of the tumor after a procedure of surgery and chemotherapy. Our research finds that the gene comprised plenty of correlations with the breast cancer, and the result may help researchers and clinicians to deeply understand the breast cancer.

TMEM family were enrolled in many pathways and functioned as the plasma membrane channel, activated signal transduction pathway, and mediates cell chemotaxis, adhesion, apoptosis, and autophagy. The research conducted by David Crottès highlighted another TMEM gene: TMEM16 A, which also played important roles in the oncogene and invasiveness of the types of cancers [2]. A mini review which was based on the TMEM88 had discovered that the TMEM88 acted as a tumor suppressor by inhibiting the Wnt pathway [3]. It could become a reality when the modern computing and technology is more intelligent and precise [4]. Kathleen Schmit et al. had found TMEM45; an inactivation of which decreased cell proliferation and modulated cell responses to cisplatin. This mechanism underlies the DNA damage repair system [5]. Choi et al. indicated that TMEM220 was a novel DNA methylation marker in human gastric cancer [6]. Numerous researchers had found that the TMEM family and their derivatives were attracting more and more attentions; the mechanism underling them had become increasingly complex and diverse [7]. However, these results indicated that TMEM65 is injected into the mitochondria and the disfunction of it may lead to the mitochondria dysfunction [8].

In our article, the TMEM65 was thoroughly advised in many databases. We mainly paid attention to its impact on expression levels, immune infiltrations, drug sensitivity, and other important markers or mechanisms (such as the TMB, MSI, and NEO). After the pan-cancer analysis, we mainly focused on its prognosis value on the breast cancer aspects. The GSEA and GSVA recognized some crucial regulatory pathways for breast cancer dominated by the TMEM65.

RETRACTED

## 2. Methods

### 2.1. Difference Analysis of the TCGA

We downloaded the original mRNA expression data and SNP data of 33 tumor data of *Pan*-cancer from the TCGA database ((for “title=”https://portal.gdc.cancer.gov/)) for further survey. Save the data which mainly contain the mRNA and SNP for the following analysis. We downloaded gene expression pattern from the GTEX database and made a combination with the TCGA database. After rectification of the data, the expression differences in genes in different cancers were calculated. The data which were downloaded from the CCLE database was also divided by the expression levels in different tissues. Additionally, the survey explores the relationship between the gene levels and the clinical stages.

### 2.2. The Analysis of Gene Expression and the Prognosis of the Cancers

Download the data from the Xena database which contained the OS and DFI for the patients from the TCGA database. Kaplan–Meier method was used for survival analysis of each cancer type (*P* < 0.05), and survival analysis was evaluated by the “survival” and “surviviner” packages. In addition, Cox analysis used “survival” and “forestplot” packages to explore the relationship between gene expression and survival.

### 2.3. Analysis of Immune Cell Infiltration

Ciberport algorithm was used to analyze the RNA SEQ data of 33 cancer patients in different subgroups, It is also used to infer the relative proportion of immune infiltrating cells and analyze the correlation between gene expression and immune cell. Additionally, the potential relationship between gene expression and immune regulatory factors (chemokines, immunosuppressants, immune-stimulating factors, and MHC molecules) was also explored through TISIDB website.

### 2.4. Drug Sensitivity Analysis

The Cellminer database is based on 60 cancer cells listed by the National Cancer Institute Cancer Research Center (NCI), and the NCI-60 cell system is currently the most widely used cancer cell population for anticancer drug research. In this study, NCI-60 drug sensitivity data and RNA SEQ gene expression data were downloaded, and the relationship between genes and sensitivity of common antitumor drugs was determined by the correlation analysis. *P* < 0.05 indicated that the results had statistical significance.

RETRACTED

### 2.5. GSVA Enrichment Analysis

GSEA analysis was used to predefine the Gene Sets, the genes were ranked well based on the expression levels in the tissues. The genes were ranked according to the expression level of the tumor tissues. In this study, GSEA was analyzed through the “cluster profiler” and “enrich blot” packages. By comparing the differences in the pathways between the high gene expression group and the low expression, we explored the possible molecular mechanism of the difference in prognosis among different patients in 33 tumors.

### 2.6. Analysis of TMB, MSI and NEO Data

TMB was defined as the somatic gene coding errors, base substitution, and total insertion or deletion mutations. In this study, the frequency of variation and the number of variants/exon length of each tumor sample were calculated. MSI values for each TCGA patient were derived from previously published studies [2] using the netmhcpan v3 0 to evaluate each patient's neoantigen [3].

### 2.7. Nomogram Model Construction

Nomogram is based on multivariate regression analysis. We used the line segment with scale and then drew them on the same plane according to a certain proportion, mainly based on the gene expression and clinical symptoms. By using those methods, we are able to distinguish the relationships between the variables in this model. Under the multivariate regression model, we scored each prognosis factor based on its impact on the survival outcomes and added all the scores of one prognosis factor to get the predictive value.

### 2.8. Statistical Analysis

All statistical analyses were performed in R language (version 4.0). The differences in the TMEM65 levels among groups were estimated using the Kruskal–Wallis test. Hazard ratios (HRS) and 95% confidence intervals were calculated using univariate survival analysis. Kaplan–Meier analysis was used to study the survival of patients based on high or low levels of gene expression. All statistical tests were bilateral (*P* < 0.05).

## 3. Results

### 3.1. Pan-Cancerous Expression Analysis of TMEM65 Gene

The expression of TMEM65 in 33 human cancers was analyzed by using TCGA and GTEX data sets. The results showed that TMEM65 was highly expressed in 24 tumor tissues; the type of the primary tumors included ACC, BLCA, BRCA, CESC, CHOL, COAD, ESCA, GBM, HNSC, KICH, LAML, LGG, LIHC, LUAD, LUSC, OV, PAAD, PCPG, PRAD, SKCM, STAD, TGCT, THCA, and UCS (Figure 1(a)). The expression level of the TMEM65 is relatively lower than that of cancer tissue. The expression of TMEM65 in different tumor cell lines in CCLE expression profile is shown in the figure. Moreover, the TMEM65 was correlated with the clinical stage of varieties of the tumors, and the tumor type comprised of BLCA, KIRC, LUSC, READ, and THCA (Figures 1(b)–1(f)). TMEM65 showed correlation with the OS for six cancers (Figures 1(g)–1(l)) and PFI for nine cancers (Figures 1(i)-1(o)). The result also established that TMEM65, which was correlated with the OS in six kinds of tumors, comprised of BRCA, LIHC, SARC, STAD, and UCEC. There was also a strong link between the TMEM65 and nine kinds of tumor types for PFI, which included ACC, BLCA, BRCA, HNSC, LGG, LIHC, PRAD, UCEC, and UVM; the KM plot consequences indicated that the TMEM65 also correlated with the KPI of the BRCA, STAD, and UCEC.

RETRACTED

### 3.2. Pan-Cancer Expression and the Immune Infiltration

As the tumor environment is composed of variety of aspect, that mainly comprise of kinds of immune mechanisms and immune cells (fibroblast, immune cells, extracellular matrix, multiple growth factors, inflammatory factor, and special cancer cells with physical and chemical characteristics). The microenvironment of the tumors played important roles in the prognosis, diagnosis, and treatment of the cancers. TMEM65 showed a significant correlation with M0 in 14 kinds of cancers, and was related with eosinophils in 13 types of cancers (Figure 2(a)). The results also indicated that TME score, CD8 T effector, and immune checkpoint scoring systems also established strong correlation with the breast cancer (Figure 2(b)).

### 3.3. Pan-Cancer Expression and Key Regulatory Genes

By using the gene coexpression analysis, we tried to explain the relationship between the TMEM65 and 33 immune-related genes: the enrolled genes were divided by the functions (such as the MHC, immunostimulating cytokine, immunosuppressive cytokine, chemokines, and chemokine receptor protein). The results showed that almost all immune-related genes were significantly associated with TMEM65 (Figures 3(a)–3(f)). Additionally, TMEM65 was strongly correlated with the some of the most common tumor-related genes and certain pathways (TGF beta signaling, TNFA signaling, hypoxia, Pyroptosis, DNA repairing, autophagy, ferroptosis, and other related genes) (Figures 3(g)–3(m)).

### 3.4. Pan-Cancer Expression for TMB, MSI, and NEO

TMB, MSI, and NEO are rising markers that showed strong correlation with the immunotherapy. The outcomes showed that the TMEM65 was strongly correlated with the TMB (OV, THCA, SKCM, and LUAD) and simultaneously indicated tight correlation with the MSI (DLBC, GBM, KIRC, and KICH). In the field of NEO, TMEM65 also indicated that it showed strong correlation with the NEO in the GBM, THCA, BRCA, LUAD, and OV (Figures 4(a)–4(c)).

### 3.5. Pan-Cancer Expression and Drug Sensitivity

Most of the patients could get a better survival prognosis after following a common procedure which mainly contained surgery and chemotherapy or neochemotherapy (Figure 5). Among all the consequences, we found that the TMEM65 showed a very strong correlation with the staurosporine, and at the same time showed negative correlation with the actinomycin D, geldanamycin analog, homoharringtonine, mithramycin, and carfilzomib.

RETRACTED

### 3.6. Pan-Cancer Expression and GSVA/GSEA

In order to explore the mechanism underlying the TMEM in a further step, we used the GSVA to cover the shortage of the GSEA. The genes were scored based on the algorithm of the GSVA. The samples were divided into high and low expression groups for further comparison by the median scores of the genes. The results indicated that TMEM65 was closely correlated with the E2F_TARGETS, G2M_CHECKPOINT, MTORC1_SIGNALING, COMPLEMENT, and MYC_TARGETS_V1 pathways. The GSEA analysis of TMEM65 for breast cancer is shown in the Figure 6.

### 3.7. Risk and Independent Prognostic Analysis of TMEM65

Nomogram prediction model was constructed according to the expression of the TMEM65 gene and clinical symptoms; the results of the regression analysis are all presented in the form of the nomogram (Figure 7(a)). Additionally, our study draws correction curves for 3-year and 5-year periods at the same time. The model was consistent with the results (Figure 7(b)).

## 4. Discussion

We had successfully confirmed that the TMEM65 was highly expressed in many types of tumors and had considerable links with the survival, immune infiltration, drug sensitivity, TMB, MSI, and NEO for many cancers. The imbalance of the TMEM65 may lead to tumorigenesis, tumoral cell proliferation, drug resistance, and other complex disorders in a large range of cancers. Among all the common tumors, breast cancer contains considerable correlations with the TMEM65. At the end of the article, we mainly focused on its impact on the breast cancer and find pathways through the GSVA/GSEA and constructed a nomogram base on the TMEM65. Above all, the TMEM65 showed tremendous correlations with most of the hot mechanisms and would be the promising research target for cancers. As mentioned above, the TMEM family genes were seldom explored deeply by the researchers. This study is the first pan-cancer analysis concerning the TMEM65 and our attention mainly lies on a variety of cancers. We hope that with the help of our findings, the researchers could understand deeper the role of the TMEM families, and design more experiments in the future.

The CCLE database provided evidence that the expression level of theTMEM65 was higher than the adjacent tissues in 24 types of cancer after analyzing a total of 33 kinds of cancers. The influence of TMEM65 on various cancers is complex and the focus of the research lies on it.

RETRACTED

OS and the PFI: for the OS aspects, we discovered that its value was more prominent in the breast cancer aspect (*P* < 0.001), the UCEC followed behind (*P*=0.0022), and the remaining cancers showed the boundary significance. We also explored the impact of the TMEM65 on predicting the clinical stage of the cancer. It is a new rising area of research, also indicates the value for the genes in evaluating the degree of malignancy of different kinds of tumors. However, there seldom exists a perfect indicating effect for the genes investigated in the current study. The pan-cancer analysis of KIF23 showed that it had a close correlation with the clinical stage and it was higher along with the higher clinical stage, but the research did not further explore the PFI and other survival index [9]. At the same time, in the research conducted by the Yun Chen, TGFBI was also elevated in various kinds of cancers (cholangiocarcinoma, colon adenocarcinoma (COAD), esophageal carcinoma (ESCA), GBM, head and neck squamous cell carcinoma (HNSC), kidney renal clear cell carcinoma (KIRC), kidney renal papillary cell carcinoma (KIRP), liver hepatocellular carcinoma (LIHC), rectum adenocarcinoma (READ), stomach adenocarcinoma (STAD), and thyroid carcinoma), and it also showed a great value in the survival aspects. While for the clinical stage aspects, it was not very obvious for the KIRC [10]. In our results, although the OS and PFI show a strong correlation for the TMEM65, the predicting value of the gene for the clinical stage was more valuable for the early stage, especially for the BLCA and THCA.

When it turns to the immune infiltration aspects, the TMEM65 was correlated with some.

Unimportant immune cells and mechanism.21 types of cancers were correlated with the T cells CD4 memory resting, and 14 types were correlated with the M0 type of the macrophage, in which 13 of them were correlated with the eosinophils. Unlike the previous similar studies, the pan-cancer research conducted by the Li et al. found that the MMP14 showed strong correlation with the six species (B cells, CD4 T cells, CD8 T cells, macrophages, dendritic cells, and neutrophils) [11]. The pan-cancer research conducted by the Bao et al. discovered that PANX1 is highly engaged in various kinds of immune cells in many cancers (CAF, macrophage, and neutrophil cells) [12]. Moreover, the survey which paid attention to the COPB1 found that for most cancers, there existed strong correlation with the immune checkpoints (BTLA, LAIR1, CTLA4, CD48, CD28, and CD200 receptor 1). However, although a strong correlation existed for the main immune-related gene, there was no significant difference in the expression of CD96 between responders and nonresponders to immunotherapy [13]. Fortunately, for our research, breast cancer showed a strong correlation with the TME score, CD8 T effector, and immune checkpoint. Lingling Bao et al. had found that all the three markers showed strong impact on the antitumor activity and an implication on the immune infiltration itself. For breast cancer, it showed a promising value for immune infiltration and the effect of immune therapy.

RETRACTED

In this study, we explored the evidence which showed the correlation between the TMB, MSI, NEO, and TMEM65. Although TMEM65 correlated with some unimportant immune-related genes, TMEM65 showed some indicative significance for the three markers for certain kinds of cancers, and the meaning behind it implies significant correlation with the prognosis of the immune therapy. At the same time, the three markers (TMB, MSI, and NEO) also attracted lots of attention in the recent similar explorations [10,11,14].

For the sensitivity for the chemotherapy aspects, the TMEM65 itself showed many implications for drug resistance. Higher expression of the TMEM65 means several chemotherapy drug resistance, and meanwhile, these results suggested that the gene could act as a promising target in overcoming multidrug resistance for the cancers. Our research is the first one that is not only concerned with the survival prognosis for the TMEM65 but also the impact for the drug resistance. Although our research successfully found TMEM65 was positively correlated with staurosporine and negatively correlated with actinomycin D, geldanamycin analog, homoharringtonine, mithramycin, and carfilzomib, the impact of the gene was weaker after comparing with similar research that paid more attention to the drug sensitivity. The research conducted by Liu et al. found that C1QTNF6 predicts a high IC50 value for most of 198 drugs which predicts drug resistance [15]. Miralaei et al. also paid attention to the drug sensitivity aspects and change in the AURKA under the presence of some chemotherapy drugs [16]. Research conducted by Zhang et al. [17]only paid more attention to XIAP and its influence on the impact of carboplatin for ovarian cancer. Therefore, our research sheds light on understanding the latent role of TMEM65 in tumor multidrug resistance and its use as a prognostic biomarker of cancers.

Our research also conducted the GSEA and GSVA research; the results also indicated that as the TMEM65 gene showed strong correlation with the cancer-related genes, higher expression of the TMEM65 means drug resistance and poorer prognosis for the breast cancer. The GSVA showed that TMEM65 was strongly correlated with the E2F_TARGETS, G2M_CHECKPOINT, MTORC1_SIGNALING, COMPLEMENT, and MYC_TARGETS_V1 pathways. The GSEA indicated that the TMEM65 gene showed strong correlation with the cell adhesion molecules, cell cycle, and oocyte meiosis, and among which the cell adhesion molecules and the cell cycle mechanisms mean a worse prognosis and higher invasive ability for cancers. E2F families are famous factors that functioned as transcription members and played dominant roles in the development of cancers. The review conducted by the Liu et al. [18]made a conclusion that the E2F family played distinct values for the breast cancer. The G2M checkpoint had become a vital marker for overcoming the metastasis of many cancers. For the breast cancer, it became the promising target for different luminal types: Oshi et al. found that G2M cell cycle pathway score can be recognized as a promising biomarker in indicating the survival for ER-positive cancers [19]. Similar research conducted by Jandial et al. made the HER-2-enriched breast cancer cells more sensitive to herceptin by inducing the G2M arrest. At the same time, the MTORC1 played multifaced roles in promoting the invasiveness of the breast cancers [20–22]. Numerous evidence also indicated the dominant role of the myc in the stemness and metastasis of the breast cancer [23–25]. The mechanisms and pathways under the analysis of the GSVA and GSEA all indicated that TMEM65 dominated several important pathways and it would be the next hotspots for the breast cancer.

RETRACTED

Overall, the shortcomings of our article are also very obvious, the impact of the TMEM65 was demonstrated in many cancers, and it seemed that the influence was more obvious for breast cancer. First of all, our research is mainly based on the public database, as a consequence of that, it lacked evidence from the laboratory data. Unlike some recent research studies, the research conducted by the Jiang et al. not only explored the function of it based on the database but also successfully demonstrated the function of the SNRPA1 for the ccRCC cells; the research successfully demonstrated that knocking down the SNRPA1 made tumor cells less invasive [26]. Similarly, the research conducted by Gao et al. had also used the same exploring pattern in the pan-cancer analysis of the PRDXs and demonstrated the pathway of the gene in the lab [27]. As a consequence, our results needed more clinical and lab data to validate in a further step, and also more related genes and pathways are needed for further validation.

In conclusion, our research successfully demonstrated that the TMEM65 is highly expressed in 24 kinds of cancers and showed a correlation with survival, immune infiltration, and recent research hotspots (pyroptosis, DNA repairing, autophagy, ferroptosis, and drug sensitivity). Moreover, we find the gene indicated more functions in the breast cancer cells and the function for the breast tumor deserved further validation in the future.

RETRACTED

## Figures and Tables

**Figure 1:** (a) The expression of TMEM65 in 33 different tumor cell lines. (b) TMEM65 was correlated with the clinical stage for the BLCA. (c)TMEM65 was correlated with the clinical stage for the KIRC, (d) TMEM65 was correlated with the clinical stage for the LUSC, (e) TMEM65 was correlated with the clinical stage for the READ, and (f) TMEM65 was correlated with the clinical stage for the THCA.TMEM65, which was correlated with the OS in six kinds of tumors, comprised of BRCA, LIHC, SARC, STAD, and UCEC (g–h) (i) The link between the TMEM65 and kinds of tumor types for PFI on forest plot. The KM curve was explored for the PFI (m–o).

**Figure 2:** (a) The correlation plot for the connection between the TMEM65 and the immune cells. (b) The TME signature box-plot for the BRCA indicated that the TMEM65 was strongly correlated with the TME score, CD8 T effector, and immune checkpoint scoring systems.

**Figure 3:** TMEM65 was correlated with almost all the immune-related genes; the genes were divided by their function ((a) MHC, (b) immunostimulating cytokine, (c) immunosuppressive cytokine, (d) chemokines, and (e)–(f) chemokine receptor protein.TMEM65 showed strong correlation with the TGF beta signaling, TNFA signaling, hypoxia, pyroptosis, DNA repairing, autophagy, and ferroptosis (g–m).

**Figure 4:** (a) TMEM65 was strongly correlated with the TMB for the OV, THCA, SKCM, and LUAD. (b) TMEM65 showed correlation with the MSI for the DLBC, GBM, KIRC, and KICH. (c) TMEM65 showed correlation with the NEO in the GBM, THCA, BRCA, LUAD, and OV.

**Figure 5:** TMEM65 was positively correlated with the staurosporine and negatively correlated with actinomycin D, geldanamycin analog, homoharringtonine, mithramycin, and carfilzomib.

**Figure 6:** (a) TMEM65 was closely correlated with the E2F_TARGETS, G2M_CHECKPOINT, MTORC1_SIGNALING, COMPLEMENT, and MYC_TARGETS_V1 pathways in the GSVA analysis. (b) The outcomes of the GSEA analysis for the TMEM65 for the breast cancer.

**Figure 7:** (a) Nomogram prediction model based on the TMEM65 level and other variables. (b) Correction curves for comparing the model and result.

## Data Availability

The data used to support the findings of this study are available from the corresponding author upon request.
